The article "circKMT2E Protect Retina from Early Diabetic Retinopathy through SIRT1 Signaling Pathway via Sponging miR-204-5p" was retracted in 2023. Reasons: signs of a paper mill; compromised peer review; unreliable results or conclusions.

# circKMT2E Protect Retina from Early Diabetic Retinopathy through SIRT1 Signaling Pathway via Sponging miR-204-5p

**DOI:** 10.1155/2022/7188193

**Published:** 2022-09-30

**Authors:** Jilai Shi, Li Li

**Affiliations:** Department of Endocrinology, The Affiliated Hospital of Shandong University of Traditional Chinese Medicine, Jinan, Shandong 250014, China

## Abstract

**Objective:**

To explore the changes of circRNAs in the retina of diabetic patients without diabetic retinopathy (DR) to screen latent protective factor.

**Methods:**

The sequencing data of the retina from three diabetic donors that possess no noticeable pathological feature of the retina at ultimate eye inspection and three healthy donative samples were involved in this study. Herein, we carried out bioinformatics analysis to disclose the expression pattern and characteristics of circRNAs on the basis of Gene Ontology as well as KEGG pathway analyses. Then, sequencing data were applied to infer the interaction between selected circRNAs and miR-204-5p. The potential miRNA response elements for the annotated circRNAs and their target gene were speculated using TargetScan as well as miRanda.

**Results:**

RNA sequencing detected 28,978 alternative circRNAs. Thereinto, 1063 were expressed with significant difference. circKMT2E was upregulated more than two folds in alloxan-induced diabetic retinal tissues compared with normal retinal tissues, exhibiting an expression trend opposite to miR-204-5p. Bioinformatics analysis showed that circKMT2E have four seed sequences on hsa-miR-204-5p. Thus, circKMT2E was speculated to have function on the basis of sponging miR-204-5p in order to participate in the pathogenetic process of DR. Besides, miR-204-5p was speculated to be able to bind SIRT1, which can interact with its target proteins, and adjusts various cell functions including cellular inflammatory responses, proliferation, as well as apoptosis.

**Conclusion:**

The upregulation of circKMT2E in the early stage of DR may be involved in its pathogenesis and may activate the SIRT1 signaling pathway to protect the retina by the sponge function to miR-204-5p.

## 1. Introduction

Diabetes mellitus (DM) as a kind of noncommunicable chronic metabolic disease has prevailed worldwide [1, 2]. The complications of DM affect nearly every tissue of the human body; among all affected tissue, diabetic retinopathy (DR) refers to the frequent microvascular complication that accompanies DM. DR currently is deemed as one of the most common causes of blindness especially in working-aged people [2, 3]. Most studies organized for western populations have found a DR prevalence of more than 30% in individuals of similar age and duration of disease [1].

In the wake of the quick progress of high-throughput sequencing approaches, the function of circular RNAs (circRNAs), which take part in significant processes in diverse diseases, has been increasingly focused on [4–7]. circRNAs, dissimilar to linear RNAs, could take shape in a closed annulus structure presenting better steadiness as well as more specific peculiarities [8–11]. circRNAs, which are normally expressed according to the stage-specific manner as well as tissue-specific pattern, can participate in a series of physiological as well as pathological processes [12–14]. circRNAs contain microRNA (miRNA) response elements, by which circRNAs could adjust the expression of their target genes [15]. circRNAs, as a type of noncoding RNAs with modulatory capacity, can weaken the impact of miRNAs on the basis of silencing miRNA via sponge function, which is related to the posttranscriptional management of genes [15, 16].

On basis of the combination of bioinformatics analysis and basic experiment, the networks of gene modulatory among mRNAs, circRNAs, and miRNAs reported by a few previous studies have offered us more profound knowledge of the process of pathology and development for the retina. Therein, miR-204, a miRNA widely expressed in the lung, kidney, eye, mammary gland, skin, as well as melanocytes, executes significant functions during both functional maintenance and retinal development [17]. miR-204, a type of enriched miRNAs in eyes, owns the most prominent expression in the ocular tissue, such as the retina, lens, and ciliary body. Therefore, the extensive expression of miR-204 implies that it could adjust several vital cellular activities for ocular tissue [18–20]. Mao et al. found that the expression levels of miR-204-5p were significantly augmented in the retina from diabetic rats; besides, miR-204-5p additionally endorses the development process of DR on the basis of downregulating the microtubule-linked protein 1 light chain 3 to inhibit autophagy [21]. However, Yang et al. found that high glucose can downregulate miR-204 in ARPE19 cells [22].

During the initial progress of DR, vascular pathology, for instance, areas of vascular nonperfusion, microaneurysms, and decreased retinal blood flow, appears [3, 23]. Reduced blood flow of the retina, to some extent, manifests inchoately, not only in humans with DM but also in animal models with DM [23, 24]. Altered accommodation of inner retinal vascular is normally deemed as an accommodation forerunner to the occurrence of grievous vascular pathology in DR [25]. The controversial capacity of miR-204 in the pathogenetic process of DR may suggest that miR-204 participates in the early protective effect but terminal disablement.

In this study, to ascertain the function of miR-204 in early diabetic retina as well as to reveal the early latent pathogenetic process of DR, in-depth sequencing data from postmortem human retinal tissue including three diabetic donors without DR and three healthy donors were enrolled. Mainly based on bioinformatics analysis, we found that the upregulation of circKMT2E in the early stage of diabetic retinal feedback may be involved in the pathogenesis of DM that activates the SIRT1 signaling pathway to protect the retina by the sponge function to miR-204-5p.

## 2. Methods

### 2.1. In-Depth Sequencing Data

The in-depth transcriptomic data of both healthy and diabetic donors (with no evident visual injury or obvious pathology of the retina at the ultimate ocular inspection) were downloaded from the NCBI BioProject database with accession numbers PRJNA672929 and PRJEB10043 using “prefetch” order in Linux with the NCBI SRA Toolkit. After stratified sampling, three healthy subjects and three diabetic subjects were signed up in this investigation. The retinal samples from a postmortem human were acquired via the Iowa Lions Eye Bank (Coralville, Iowa, USA) in which samples were safeguarded within 6 h postmortem [26]. For the option of donors, Becker et al. [26] did not enlist donors who possess a confirmed medical history of Hepatitis B or C and HIV. Besides, donated ocular samples that were provided with neurodegenerative diseases were also excluded.

### 2.2. Differential Gene Expression Analysis

Sequencing reads with satisfying quality were matched to the online reference genome or transcriptome with the aid of STAR software (v2.5.1b) [27]. All identified circRNAs on the basis of DCC software were then annotated with the aid of the circBase database as well as Circ2Traits. circRNAs that possess significant differential appearance between the above-mentioned two groups were recognized based on *t*-test. The *p* value was corrected using the Benjamini and Hochberg method [28]. Fold change ≥ 2.0 as well as *p* value ≤ 0.05 were used for filtering circRNAs with differential expression.

### 2.3. Enrichment Analyses on Basis of GO and KEGG

Enrichment analyses on the basis of GO (http://www.geneontology.org) as well as KEGG (http://www.genome.jp/kegg) were implemented on the host genes of circRNAs with differential expression. GO is a methodic and organized database in order to depict both genes and its product. It not only covered molecular function but also revealed biological processes as well as cell component. With the help of the pathway analysis from KEGG, the signaling pathways that contain circRNAs as well as their biological functions can be inferred. The relevant *p* value was computed on the basis of Fisher's exact test, with a suggested threshold value at 0.05.

### 2.4. Early DR-Related Candidate circRNA Analysis

The abundance of circRNAs was calculated by Ballgown and computed by Fragments Per Kilobase of exon model per Million mapped fragments (FPKM). The threshold value of FPKM in each group was 0.5, which mean the circRNA would be deemed as expressing in this group if FPKM > 0.5. For the circRNA expression, Student's *t*-test was applied on the basis of GraphPad Prism 8.0 to compute the significance for differences.

### 2.5. Interaction Network Analysis of circRNA, miRNA, and Target Gene

The underlying miRNA reaction elements for the annotated circRNAs and target gene were predicted using custom-written software on the basis of both TargetScan and miRanda (Cloud-seq Biotech, Shanghai, China). CircPrimer1.2 (http://www.bioinf.com.cn/) and UCSC genome browser were used to annotate the arrangement of circKMT2E and its positions on parental genes, respectively. circMir1.0 software, on the basis of miRanda 2010 (http://www.microRNA.org/microRNA/getDownloads.do) and RNAhybrid-2.1.2 (https://bibiserv.cebitec.uni-bielefeld.de/rnahybrid/), was applied to annotate putative bundling situations of miR-204-5p on circKMT2E transcripts.

## 3. Results

### 3.1. Overall Result of RNA Sequencing

We identified the expression level of numerous circRNAs existing in retinal tissues on the basis of the samples donated from the diabetic subjects with no conspicuous visual damage or observable pathology at ultimate ocular detection as well as the retinal tissues from control healthy donors using the high-throughput sequencing. Under the sequencing, a total of 28,978 circRNAs were perceived in human retinal tissues, of which 10,970 circRNAs were observed for the first time as newfound circRNAs, while 18,008 circRNAs were already included in the circBase. (Figure 1(b)). According to the functional explanation in this study, which refers to the genome of these annotated circRNAs, 75.09% of these circRNAs were situated in protein-coding exons, while 0.69%, 1.24%, 6.11%, and 16.87% of them belonged to introns, intergenic, antisense, and sense overlapping regions, respectively (Figure 1(a)). The median size of exonic circRNAs was distributed at 556 nt (Figure 1(c)).

### 3.2. Expression Pattern and Characteristics of circRNAs in Retinal Tissues in Type 2 Diabetes Patients without Diabetic Retinopathy

Differentially expressed circRNAs between above-mentioned two groups are exhibited on the basis of a scatter plot (Figure 2(a)). As shown in the volcano plot (*p* ≤ 0.05 as well as fold change ≥ 2.0), the number of 1063 circRNAs was disclosed to present significant differential expression between the above-mentioned two groups, of which 142 circRNAs were increased and 921 circRNAs were decreased in the DM group in contrast with the control group (Figure 2(b)). Among screened circRNAs with differential expression, 198 circRNAs were detected as novel circRNAs, and 865 circRNAs were already included in the circBase (Figure 2(c)). Besides, a total of 14 circRNAs were revealed to present more than 5-fold differential expression, including circMET, circITCH, circDNMT3B, circPAG1, circADAM9, circFTO, circ001209, circKMT2E, circCOL1A2, circ0001953, circHIPK3, circ0084043, circZNF532, and circEhmt1 (Figure 2(d)).

### 3.3. Distribution of the circRNAs with Differential Expression

Among 1063 differentially expressed circRNAs, 1056 were derived from 805 unique genes, while the host genes of 7 circRNAs cannot be ascertained. 81.49% of the 805 genes generated only one circRNA, 11.80% of these genes generated two different circRNAs, and 6.71% of these genes generated more than two circRNAs (Figure 3(a)). In addition, these circRNAs differentially distributed throughout all of human chromosomes (Figures 3(b) and 3(c)).

### 3.4. Gene Ontology and KEGG Pathway Analyses of Differentially Expressed circRNAs

In the process of bioinformatics analysis, to annotate the capacity of the target genes of all circRNAs that were differentially expressed, Gene Ontology analysis was applied. The top ten enriched functional entries of cellular components, biological processes, and molecular functions are shown in Figure 4. The most enriched biological process was intracellular metabolic, organelle organization as well as cell protein metabolic process (Figure 4(a)). Of the cellular components, the genes were closely related to the intracellular part, intracellular organelle, cytoplasm, and catalytic complex (Figure 4(b)). For the molecular functions, the largest proportion of top genes was referred to as binding and protein binding (Figure 4(c)). To further understand the correlation between these top genes and the pathogenesis of the early DR, we employed pathway analysis based on KEGG. The top ten strikingly enriched KEGG pathways are shown in Figure 4(d).

### 3.5. The Latent Connection between miR-204-5p and circRNA

Due to the specific significance of miR-204 in the biology of the retina [17, 22], in this study, what circRNAs the predicted miRNA targets were identified on the basis of miRNA target prediction software—TargetScan. A total of 240 circRNAs were inferred to possess miR-204-5p response elements. By comparing these circRNAs with the differentially expressed genes in DM retina, our research team discovered that 206 (85.83%, 206/240) circRNAs were expressed with significant difference in the DM group, including 18 (7.5%, 18/240) upregulated and 188 (78.33%, 188/240) downregulated circRNAs (Figure 5(a)). That is, the alteration of the miR-204-5p-related circRNAs seems to be associated with the pathogenesis of DM.

The predicted mutual combination of miRNA and circRNA was ranked according to pairing structure scores computed by miRanda algorithms, with the result revealing that hsa-miR-204-5p had a high score for upregulating circRNA circKMT2E and downregulating circRNA circPAG1. Hence, circKMT2E and circPAG1 were further used for the FPKM analysis. These two circRNAs both showed the same expression patterns with the sequencing results (Figure 5(b)). circKMT2E is upregulated significantly (FC = 4.449, *p* = 0.047), while circPAG1 is downregulated significantly (FC = 0.413, *p* = 0.021), in the DM group in contrast to the healthy control.

Besides, circKMT2E, derived from Exon4-Exon15 of transcript KMT2E of Chromosome 7 (q22.3) (Figures 6(a) and 6(b)), was significantly upregulated in DM retina and exhibiting an opposite expression pattern to miR-204-5p. Bioinformatics prediction revealed that circKMT2E having four matched sequences could combine with miR-204-5p (Figures 6(c) and 6(d)). Further analysis of TargetScan revealed that miR-204-5p could combine with SIRT1. Briefly, circKMT2E seems can activate the SIRT1 signaling pathway by the sponge function to miR-204-5p.

## 4. Discussion

circRNAs and miRNAs, which have dynamic and tissue- and cell-type-specific expression patterns, attract many researches to focus on their potential function, especially on their roles in the pathogenesis of diseases and the possibility to serve as fresh therapeutic targets for DR treatment [29]. Currently, most general studies show that circRNA can frequently act as the “sponges” of correlative miRNA and decrease the inhibiting effect of miRNAs toward target gene expression [28, 30]. In this study, compared with the control group, 14 different circRNAs in retinal samples from diabetic donors who do not possess conspicuous ocular impairment or obvious pathology of the retina at the last eye exam were revealed to present significant alteration and may participate in the early pathological feedback of DR. Some of this circRNAs have been confirmed by systematic research; for example, Zhu et al. [31] found that downregulation of circDMNT3B was conducive to the vascular dysfunction of DR on basis of targeting miR-20b-5p and BAMBI (a type 1 TGF*β* receptor antagonist), and Shan et al. [32] found that circZNF532 adjusts diabetes-induced retinal pericyte deterioration as well as vascular dysfunction.

It was reported by Qi et al. [21] as well as Yang et al. [22] that miR-204 may be significative in the pathogenesis of DR; however, both the capacity of miR-204 in the early phase of DR and its upstream mechanism are remain sealed. Thus, we launched this study by focusing on miR-204. Based on RNA-seq and FPKM analysis as well as a previous study of miR-204-5p, we further focused on circKMT2E, which is derived from the fourth to fifteenth exons of the annotated KMT2E gene region. circKMT2E was significantly upregulated in diabetic donors without DR and showed a conflicting expression pattern to miR-204-5p. Bioinformatics analysis further revealed that circKMT2E possesses four seed sequences that can be matched with hsa-miR-204-5p. Thus, we deduced that circKMT2E, to some extent, may be a potential controller in the early pathological process of diabetic retina and be associated with the miR-204-5p sponge function. Same as the previous study conducted by Lv et al. [33] that focused on islet *β*-cells, our bioinformatics analysis showed that human miR-204-5p can bind SIRT1.

KMT2E is usually related to neurodevelopmental diseases, such as autism spectrum disorder, mental retardation, macrosomia, neurodevelopmental disorders, and epilepsy [34, 35]. Thus, since the retina contains abundant neuronal quantity and separate neuronal types [36], the circKMT2E seems to broadly benefit diabetic retina. Besides, miR-204 was also previously described to have various regulatory functions such as serving as an autophagy- and apoptosis-related controlling factor in various diseases. Besides, Yan et al. reported that the ischemia reperfusion injury of the spinal cord can be protected on the basis of the inhibition of miR-204, which is possible with the aid of promoting autophagy and antiapoptosis [37]. Jian et al. disclosed that miR-204 protected cardiomyocytes by adjusting autophagy through regulating LC3-II protein during hypoxia reoxygenation, and Cheng et al. [38] found that endogenous miR-204 can protect the kidney against chronic injury in hypertension and diabetes. That is, miR-204 can present diverse function for different tissues. In addition, Qi et al. found that miR-204-5p was presented as considerably augmented in the retina tissue collected from diabetic rats and further found that miR-204-5p can promote DR development [21]. However, Yang et al. found that high glucose can downregulate miR-204 in ARPE19 cells, which is a kind of human retinal pigment epithelial cell line [22]. It seems that miR-204-5p has both a stage- and a tissue-specific manner.

SIRT1, a constituent of the silent information regulator 2 family, is a Class III histone deacetylase, which interplays with target proteins, and adjusts many cellular progresses, for example, cellular apoptosis, proliferation, and inflammatory responses [33, 39]. Generally, Sirt1 is mainly a histone deacetylase predominately localized in the nucleus, and its activity relies on cellular NAD availability [39]. Functionally, SIRT1 could deacetylate a series of histones, for example, H3 and H4, and more than 50 transcription factors and DNA repair proteins, for example, NF-*κ*B [40]. It is expressed throughout the retina and is currently deemed as a guardian of the development of DR. In addition, the associative ability of miR-204-5p to SIRT1 was confirmed by a previous study [41]. Thus, in the early stage of diabetic retinal feedback, the upregulation of circKMT2E may be involved in the pathogenesis of DM on the basis of activating the SIRT1 signaling pathway to protect the retina by the sponge function to miR-204-5p, just as the augment of Sirt1 is also defensive against diverse ocular diseases such as cataract, retinal degeneration, as well as optic neuritis [39, 42].

Therefore, this study substantially appended to previous studies by finding that, in the early stage of diabetic retinal reaction, circKMT2E can seemingly activate the SIRT1 signaling pathway to defend the retina based on its sponge function to miR-204-5p. Besides, this study illustrated the controversial capacity of miR-204-5p in early diabetic retina. However, this study possesses several limitations. First, the direct binding abilities of circKMT2E and miR-204-5p were not substantiated by dual-luciferase reporter assay. Second, the transfection experiment of the retinal cell was not included in this study. Third, which factor makes miR-204-5p lose efficacy and induce DR was not ascertained. Although our study found that the differentially expressed circRNAs were involved in the pathologic process of DR and offered an innovative target for the therapy of DR, the exact mechanisms need further validation.

## 5. Conclusion

In the present study, our research team scrutinized the circRNAs that possess differential expression in the retina from diabetic donors who did not possess ocular damage or retinal alteration of pathology and preliminarily discussed the relation between miR-204-5p and related circRNAs during the early diabetic retina. The upregulation of circKMT2E in the early stage of diabetic retinal feedback may be involved in the pathogenesis of DM that activates the SIRT1 signaling pathway to protect retina by the sponge function to miR-204-5p.

## Figures and Tables

**Figure 1:** Overall result of RNA sequencing. (a) The genomic location of circRNAs. (b) The amount of circRNAs as well as their junction reads discerned in DR as well as normal tissues. (c) The length distribution of exonic circRNAs.

**Figure 2:** Differential expression of circRNAs in diabetic retinopathy tissues. (a) The scatter plot of circRNA expression of the retinal tissues from diabetes mellitus (DM) and control groups. The middle black line indicates that the DM and normal control groups present no significant difference. circRNAs beyond the top black line or under the bottom black line signpost >2-fold alterations. The red spots disclose augmented circRNAs, and the green spots reveal diminished circRNAs in the DR group in contrast to the control group (fold change ≥ 2.0). (b) The volcano plot of the circRNAs with remarkable differential expression between two groups. The vertical green lines represent 2.0-fold (log2 scaled) augmented and diminished changes. The horizontal green line refers to a *p* value of 0.05 (−log10 scaled). The red spots represent circRNAs with remarkable differential expression (fold change ≥ 2.0, *p* ≤ 0.05). (c) A number of 1063 circRNAs are significantly differentially expressed with ≥2-fold changes (*p* ≤ 0.05) in the DM group in contrast to the control group. There are 142 significantly upregulated circRNAs and 921 significantly downregulated circRNAs, including 198 novel circRNAs (red). (d) A number of 1063 circRNAs were probed to having a significant changed expression between two groups, and 14 circRNAs that presented more than 5-fold difference were delivered in this figure. The circRNAs with high expression were red-colored, while circRNAs with low expression were green-colored.

**Figure 3:** Distribution of the differentially expressed circRNAs. (a) Analysis of circRNAs and their host genes shows most genes (81.49%) generating only one circRNA. (b) Chromosomal distribution of the differentially expressed circRNAs. (c) Chromosomal distribution of screened circRNAs in the human chromosomes. The farthest outer layer discloses the situation of the circRNAs. From the outside to the inside, the inner circles disclosed the expression distribution of all circRNAs in diabetic as well as normal samples.

**Figure 4:** Gene ontology analysis as well as Kyoto Encyclopedia of Genes and Genomes analysis of the host genes of circRNAs with differential expression. GO analysis annotates differentially expressed circRNAs through three aspects, including (a) biological process, (b) cellular components, and (c) molecular function. The bar plots show the top ten improvement score values of the expressive enrichment terms. (d) The top ten relevant pathways are identified for the differentially expressed circRNAs. The enrichment score value of displayed Pathway ID equals “−log10 (*p* value).” The dot plot discloses the top ten enrichment score (−log10 (*p* value)) values of the expressive enrichment pathway.

**Figure 5:** Screening the miR-204-5p binding circRNAs and validating their expression pattern by FPKM analysis. (a) An overlapping number of miR-204-5p binding circRNAs and differentially expressed circRNAs in DM and control retina (DM-up: upregulated circRNAs in diabetic retinopathy; DM-down: downregulated circRNAs in diabetic retinopathy). (b) Validation of circRNA expression by FPKM analysis. Bars represent mean ± SEM (^∗^*p* < 0.05; DM: diabetic cataract; FC: fold change). ^∗^*p* < 0.05.

**Figure 6:** It seems circKMT2E can activate the SIRT1 signaling pathway by the sponge function to miR-204-5p. (a) The structure of circKMT2E located between the fourth and fifteenth exons of the KMT2E gene. (b) The assumed binding sites of miR-204-5p on circKMT2E. (c) Detailed annotation of the predicted binding site sequence between circKMT2E and miR-204-5p. The “2D Structure” column displays the combining sequence of circKMT2E and miR-204-5p. The “Local AU” shows the upstream and downstream of 30 nucleotides of the seed sequence. The “Position” column exhibits the possible situation of miRNA response elements on circRNA sequence. (d) miR-204-5p possesses binding site for SIRT1.

## Data Availability

The labeled dataset used to support the findings of this study are available from the corresponding author upon request.
